# Improved Artificial Neural Network with State Order Dataset Estimation for Brain Cancer Cell Diagnosis

This article has been retracted.

**DOI:** 10.1155/2022/7799812

**Published:** 2022-04-16

**Authors:** D. N. V. S. L. S. Indira, Rajendra Kumar Ganiya, P. Ashok Babu, A. Jasmine Xavier, L. Kavisankar, S. Hemalatha, V. Senthilkumar, T. Kavitha, A. Rajaram, Karthik Annam, Alazar Yeshitla

**Affiliations:** ^1^Department of Information Technology, Seshadri Rao Gudlavalleru Engineering College, Gudlavalleru, Andra Pradesh, India; ^2^Department of Information Technology, Vignan's Institute of Information Technology, Visakhapatnam, Andra Pradesh, India; ^3^Department of Electronics and Communication Engineering, Institute of Aeronautical Engineering, Dundigal, Hydrabad, India; ^4^St. Xavier's College (Autonomous), Palayamkottai, Tamil Nadu, India; ^5^Department of Computer Science and Engineering, SRM Institute of Science and Technology, Chennai, India; ^6^Department of Computer Science and Engineering, Panimalar Institute of Technology, Chennai, India; ^7^Department of Electronics and Communication Engineering, Megha Institute of Engineering & Technology, India; ^8^Department of Computer, Applications, Kongu Engineering College, Perundurai, India; ^9^Department of Electronics and Communication Engineering, EGS Pillay Engineering College, Nagapattinam 611002, India; ^10^Department of Biotechnology, College of Biological and Chemical Engineering, Addis Ababa Science and Technology University, Ethiopia

## Abstract

Brain cancer is one of the cell synthesis diseases. Brain cancer cells are analyzed for patient diagnosis. Due to this composite cell, the conceptual classifications differ from each and every brain cancer investigation. In the gene test, patient prognosis is identified based on individual biocell appearance. Classification of advanced artificial neural network subtypes attains improved performance compared to previous enhanced artificial neural network (EANN) biocell subtype investigation. In this research, the proposed features are selected based on improved gene expression programming (IGEP) with modified brute force algorithm. Then, the maximum and minimum term survivals are classified by using PCA with enhanced artificial neural network (EANN). In this, the improved gene expression programming (IGEP) effectual features are selected by using remainder performance to improve the prognosis efficiency. This system is estimated by using the Cancer Genome Atlas (CGA) dataset. Simulation outputs present improved gene expression programming (IGEP) with modified brute force algorithm which achieves accurate efficiency of 96.37%, specificity of 96.37%, sensitivity of 98.37%, precision of 78.78%, *F*-measure of 80.22%, and recall of 64.29% when compared to generalized regression neural network (GRNN), improved extreme learning machine (IELM) with minimum redundancy maximum relevance (MRMR) method, and support vector machine (SVM).

## 1. Introduction

This research work presents the static and static-order dataset based on enhancing artificial neural network for classifying glia blastemal multiform state [1]. This classification segment is used for diseased cell predicting the purpose for dynamic-order cancer cell growth in the brain. Hundreds of genes were chosen, and a 10-gene profile was recognized as a predictor. If a brain tumour is detected, your doctor may offer a variety of tests and procedures, including the following:

- An examination of the nervous system. A universal testing machine may entail testing the sight, audio, balancing, cooperation, stamina, and reactions, among many other things. Difficulties in one or more regions could indicate which section of the brain is being damaged by something like a brain tumour
- Radiology tests are performed. Head cancers are frequently diagnosed with magnetic resonance imaging (MRI). Throughout your MRI study, a dye may be put into a vein in your arm

The presented research work is focused on the research restricted factor of the glia blastemal multiform (GBM) datasets from the TCGA. A blend of numerous data types is huge and redundant, which will root a computational crisis. Choosing an appropriate classifier is also a harsh mission for the removal of not number terms. Research paper explains about the benefits of both feature reduction technique and classification technique. Initially, feature reduction technique is used to improve gene expression programming. Next, brute force algorithm which has algorithm level concept, and then enhanced artificial neural network (EANN), is used for classification process [2, 3]. The EANN (enhanced artificial neural network) is popularly used in the diagnosis of cancers. It includes treating various types of cancers like glia blastemal multiform cancer, lung cancer, colorectal cancer, and prostate cancer. Also, by using the cell shape data, it performs differentiating the extremely aggressive cancer cell lines from the normally invasive cancer cell lines [4]. The EANN is also been used for the acceleration of the analysis of dependability for the organizations subjecting to expected disasters and to forecast the groundwork expenditures [5]. In this research work, a brief study on the improvement of the accuracy levels is projected and compared with the previous works. The success of radiomics relies upon the essential factors like accuracy, greater reliability, and high efficiency of the prognostic and the predictive flow. Consequently, the radiomics-centered medical biomarkers fundamentally require the comparison of various supervised learning approaches. The proposed research work is an improved supervised learning method for both improved gene expression programming and enhanced artificial neural network classification method. A unique way used for brain cancer diagnosis prediction replica is to enhance the medical therapy instructions and to find the affected area where the disease affected the person's life [6]. In recent survey, cancer cell prognosis has various techniques to predict the disease-affected region.

This proposed work is summarized as follows: Section 2 is the literature survey related to this proposed method.  Section 3 describes the proposed methodology and various algorithms are given.  Section 4 is the performance evaluation analysis.  Section 5 is the result and discussion.  Section 6 concludes the overall methodology used.

## 2. Literature Survey

Kim [2] has presented the pipeline-channeled quickening architecture for allay maximum computing order of an ANN (artificial neural network). It is specifically an RBM-based ANN. RBM is the restricted Boltzmann machine ANN. It provides computational achievements with connection updates of around three hundred billion per second and it shows a faster achievement rate; i.e., it is 193 times faster than the software-enabled solution from the all-purpose processors. Also, this architecture showed a four times faster process than the previous performances.

Cortes et al. [1] have proposed a unique technique for adaptively learning artificial neural networks. It is the theoretical analysis with the generalization of data dependency with the proof of efficiency and discussion on the future works which were dealt. End up of industrial observation with one of the techniques with different duo grade works is extracted from the CIFAR-10 dataset. End up explains that the technique can automatically study the network structures, with each aggressive work accuracy relating to the accomplished classic way findings for the neural networks.

Song et al. [7] have proposed CBTM (continuous body temperature measurement) which is the greatest implication for observing the health of human beings. The noninvasive wearable thermometers involved in the CBTM circumvent the interference with the regular routine activities of the users. Therefore, the wearable and noninvasive thermometers operate with the steady-state models and end up of this experiment takes huge time and is physically disturbed by the user's movements. Yet, there is no way to solve the problems that occurred. In this model, wearable and the nonwearable temperature difference is calculated. Next, the link between the temperatures, the skin, and the human body is analyzed using ANNs. Finally, this novel explains the multiple artificial neural networks based on the CBTM technique. This proposed model exhibited that the reaction time is one to ten compared to the other common CBTM approaches which is wearable noninvasive exhibiting high accuracy and high stability.

Zhao et al. [8] have presented an artificial network-assisted IA approach with the feature of WPT (wireless power transfer). Here, the artificial network was created by data streams of each of the transmitters that provide interference-free rattle of the snooping process. This work also touches on the fact that the efficacy of energy harvesting and security is not a determining factor of the transmitter power in artificial networks. The total transmitted power of the artificial network is increased in order to function the antisnooping. It is achieved by involving the optimization of the power transmitted and the power split coefficient with the need of SINR (signal interference noise ratio) and satisfies the power collection. The derivative analysis of the closed solutions resolves these issues with minimum computational difficulties. End up has explained the effectiveness of the improved technique.

Elkatatny et al. [3] have exhibited that the methodical machine learning of the wave function would reduce the intricacy of the manageable simulational model, rarely for physical notice. This work explains the representation variation of the quantum state development based on the ANNs with a varying amount of invisible neurons. It discusses the complications of the quantum systems by applying the corroboration learning method, whereas, ground state finding capacity or unitary time progresses. Thus, relatively higher accuracy of the dynamical and the equilibrium dimension and properties of the prototype interaction spin model serves as an effective tool for resolving the quantum multibody problems.

Sharma et al. [5] have proposed the many bandwidth-constrained objective SBMAP (segmented brute force mapping approach) algorithms to serve optimum energy efficiency and less complex computations for the patterned NoC. This algorithm provides embedded system mapping onto the NoC system processing elements effectively and distributes the application to several segments. These properties are used for the modern methodical search protocols that exhibit advanced simulation time and enhanced performance. The state-of-the-art techniques like the near-optimal mapping, the branch and bound mapping, and the random mapping approaches were compared with the SBMAP algorithm that maps the workload of the real-time applications. The result of the proposed system is more effective than the existing algorithm.

Carleo and Troyer [9] have proposed the RSA cryptosystem for security which equals the modulus size, *n*, where *n* is the multiple of any two largest prime numbers, denoting it as the variables *p* and *q*. The variable *n* is a public cryptanalyst which is used in the factorization approaches such as Pollard's technique and Euler's method for calculating the private keys *p* and *q*. The functions of this brute force technique include the generation, evaluation of possible solutions, and verification of such candidate solutions which one by one agreed to discover the finest solution. The random search technique is the numerical optimization method, which initializes the search process with one candidate solution generation aimlessly to find the best effective solution. This works explains the pros of the brute force algorithm and random search technique to enable effective factoring of RSA modulus via Python language and test on optimality using Fermat algorithm.

Verma et al. [10] have designed a wearable AAC device (augmentative and alternative communication). It supports the communication of the paralysis sufferers, by converting the distinct breathing patterns into the predefined words. They found these recordings of the breath signal into the strong and the soft blows to produce discontinuous breathing patterns. This study works on the paralysis sufferer of a certain age bar with active emotional functionalities. This work has no threshold limit to set a stable condition to organize the breathing signal into the soft blow and the strong blow. Each person has a different amplitude of the soft blow and the strong blow; it is based on the statistical exam that generates greater deviance and overlapping signals without any threshold limits. Thus, an algorithm is proposed using the concept of the brute force algorithm. This new algorithm requests the user to set the threshold limits during initialization, wherein the limits of the input were given as the soft breath and the hard blow. Thus, the device's accuracy is derived with the values of the standard error of the mean, and value score was 15.45 ± 0.1141 out of 16.

Khan et al. [11] have investigated predicting the impending performance of the present network that is modeled. The inverse effects were resolved by genetic software design. Similarly, gene expression software design contributes to discovering real differential system model. The inverse effect issues of the ordinary differential equation are resolved by this novel approach. This model may control the diversity and speed up the technique. This model has improved the techniques to work on time efficiency and better precision prediction than the existing traditional approaches.

Milukow et al. [12] have introduced an algorithm of GEP (gene expression programming) for measuring the TBM with respect to the penetration rate. The GEP model database consists of about seven model inputs regarding the characteristic properties of the machine and output as the penetration rate. The multiple regression method understands the overall capability of the algorithm. A series of work ratios were analyzed to opt for the best possible GEP and MR equations. The system results of the gene expression programming equation established on the *R*_2_ (coefficient of determination) were estimated to be 0.855 on training and 0.829 on testing datasets, wherein the proposed MR equation showed 0.795 and 0.789, respectively. This work suggested that the gene expression programming equation is more effective and this generates the new equation for prediction work in TBM.

Armaghani et al. [13] proposed a novel technique in the direction of predicting mechanical properties of the RAC (recycled aggregate concrete) by using the GEP method. An enormous predictable test database consists of the end up around 650 compressive strength, the elastic modulus of around 421, the splitting tensile strength of 346, and the flexural strength of 152; the tests of nonpozzolanic commixture RACs were analyzed through the review survey. The selected statistical indicators explain the end up appraisal, and the database provides the traditional RAC model's mechanical properties. With this database, new expressions were framed to predict a 28-day splitting tensile strength, the elastic modulus, the strength, and the flexural weightage of RACs. Results and analysis sections stated that the calculated end up showed better prediction capability with the test end up. And this design also showed enhanced mechanical property measurement than all other existing methods.

Sabar et al. [14] have proposed a novel advanced strategy for the enhanced hyperheuristic framework. This work utilizes dynamic multiple-armed bandit extremities for selecting the suitable heuristic model realistic for every implementation. Additionally, they also proposed the GEP framework, which executes the approval benchmark of individual issue automatically in detail, rather than using human-designed criteria. The generalization of the proposed work is explained by the combinational optimization issues: one static and one dynamic. Upon comparing the results of the popular acceptance benchmark, bespoke methods, and the other hyperheuristic models, the projected end up stated that the proposed work establishes both the domains. Further comparison was made with the hyperheuristic competition (CHeSC) test suite for performance analysis.

Nag et al. [15] have proposed a unified algorithm for simulating the FS (feature selection) and the structure of the diversity that classifies the utilization of a steady-state multiple-objective GP (genetic programming) that reduces the occurrence of the FN (false negative), the FP (false positive), and the number of leafy nodes on the tree. This proposed work splits the *c* class issue into the *c* binary taxonomy issues. The *c* sets of genetic programs were expanded to create the *c* band. In the alteration process, the fitness and the unfitness of features were achieved, which modifies dynamically with reproduction to highly related features with less repetition. The proposed work is compared with the biobjective GP model which does not utilize any of the rule size decrease and the FS strategy. They also illustrated the performance of the FS model and the rule size reducing model.

Lv et al. [16] have proposed a probabilistic assessment method. In this, the brake pressure is created for the EV vehicles centered with the multilayer ANN (artificial neural network) that uses the training technique LMBP (Levenberg-Marquardt backpropagation) training technique. Initially, the advanced architecture of this proposed multiple-layered ANN applied for the brake pressure evaluation was discussed. Then, the standard BP (backpropagation) technique trains the FFNN (feedforward neural network). An effective training technique of the LMBP process was developed based on the BP concept. Secondly, the frame dynamometer under the standard driving cycles carried the testing process of the real vehicle. The resultant data of the power train and the vehicle systems were collected and analyzed, and the featured trajectories for the FFNN train collections were predicted. Finally, measured vehicle data-enabled training produced multiple-layered ANN and calculates the work of the brake pressure appraisal and related it with other existing learning approaches. End up showcased excellent feasibility and the rate of accuracy in the projected ANN-based technique pressure braking evaluation on the original delay mechanism.

Yousefzadeh et al. [17] have been concerned about the recent advancements of event-based vision sensors. The creative technologies are used by new researchers and highlight such advanced sensors and their potential to exhibit a very low-latency sensing rate rapidly. The power efficiency, dynamic range, data compression, and temporal resolution of these sensors exceed the frame-based vision sensors. Yet, the ANN and the SNN (surpass spiking neural networks) showed high accuracy rate acceptance. The exploitation of the event-based and frame-based processing techniques was achieved via this work. They utilized FPGA and MNIST datasets for designing the network. They also provided the HDL codes.

Table 1 shows the comparison of pros and cons for different algorithms.

## 3. Proposed Methodology

The recognized dominant features of the proposed model produced higher arrangement accuracy and minimize the missed detection and the false alarm rate than the existing feature classification. The specific features of the selection and classification were analyzed in this proposed work.

The predictive model for the clinical results is accounted for both the conditions within and in between the platform interactions of the IGEP (improved gene expression programming). The proposed approach tested with the simulated datasets. The results indicated that it estimates the feature sets efficiently. Concurrent measurements of genetic and epigenetic characteristics illustrated the functions of their complex relationships played in the disease progression and outcomes. The projected algorithm processes are provided in Figure 1.

### 3.1. Dataset Configuration

This dataset collection is selected from previous research work. The dataset is given in Table 2.

Datasets consist miRNA expression, gene copy number, gene methylation, gene expression, and disease-affected human age at estimation that were repossessed from original data for further technique. In our model, age is a stable measurement of a critical factor in brain cancer cell prognosis. Classification of our listed dataset is presented in Table 2.

Static properties of dataset concepts are presented in Table 3. Based on these datasets, the proposed method is modeled.

### 3.2. Improved Gene Expression Programming (IGEP)

The best recognized supervised method is improved gene expression programming (IGEP), which aspects for protrusion directions on which the ratio of the between-class covariance to within-class covariance is exploited. Based on the prediction techniques, there arise three critical problems.

- Problems involving numeric (continuous) predictions
- Problems involving categorical or nominal predictions, both binomial and multinomial
- Problems involving binary or Boolean predictions

The first type of the problem goes by the regression name and then the organization through logistic deterioration as a superior situation. Also, the crispy organizations “Yes” and “No” likelihood committed with the individual results and then associated with the Boolean algebra and fusion logics. The confusion matrix parameters are given in Figure 2.

### 3.3. Brute Force Algorithm

The brute force algorithm is considered as the checking protocol at all the positions on the text between the zero and *n*-*m* positions; the initialization of the occurrence of the pattern is monitored. The pattern is shifted to one next position to the right by the BF after both attempts. This algorithm does not require continual space along with the text and the pattern, and also, no preprocessing stage is required. This is one of the main features of the brute force algorithm. The comparison of the character text can be done in random order in the searching period. The predictable count of text character evaluations equals 2*n*.

The presented approach utilized accuracy improvement in our proposed method.

### 3.4. Enhanced Artificial Neural Network (EANN)

The proposed EANN (enhanced artificial neural network) involves the short-term behavior models of each neuron, the model predicting the rise of the changing aspects of the neural circuitry from the communications among neurons, and at last, how the model behaviors arose from the intellectual neural modules which signify the completion of the subsystem. The models of the durable and interim plasticity of the neural networks and links to learn and the memory after each neuron to the system are included. In the static regression, it follows the static approach to model the association among the scalar response, i.e., the dependent variables, and one or more explanatory variables, i.e., the independent variables. The simple static regression exhibits one explanatory variable. The multiple static regressions exhibit more than one explanatory variable. The static predictor functions are used to model the static regression relationships, whose unidentified model parameters are projected from the data.

The dataset is presented in order of{*b*_*i*,_*a*_*i*1,⋯,_*a*_*ip*_}_*i*=1_^*n*^, where *n* is the static units, *p* is the vector of repressors, and *x* is static. Unobserved random numerical order that includes “noise” to the static relationship between the dependent numerical patterns takes the term from *b*_*i*_:

(1) $$\begin{array}{c} b_{i}=\alpha_{01}+\alpha_{1}\alpha_{i1}+\cdots \alpha_{pxip}+i={a_{i}}^{\text{T}}\alpha +i,\;i=1,2,\cdots ,n, \end{array}$$

where *T* is considered as the transpose; therefore, *a*_*i*_^T^*α* is the inner product between vectors *x*_*i*_ and *α*. *N* equations are stacked together and written in matrix documentation as follows:

(2) $$\begin{array}{c} b=a\alpha +\in , \end{array}$$

where

(3) $$\begin{array}{c} b=\left(\frac{y_{1}}{y_{2}..y_{n}\;}\right), \end{array}$$

(4) $$\begin{array}{c} a=\left(\frac{a_{1}^{T}a_{2}^{T}\cdots }{a_{n}^{T}}\right)=\left(\frac{1a_{11}\cdots a_{1p}1a_{21}\cdots a_{2p}}{::1a_{n1}\cdots a_{np}}\right), \end{array}$$

(5) $$\begin{array}{c} \alpha =\left(\frac{\alpha_{0}}{\alpha_{1}\alpha_{2}\cdots \alpha_{p}}\right),\in =\left(\frac{\in_{1}\;\in_{2}.}{..\in_{n}\;}\right), \end{array}$$

where *a* is the independent variable and *b* is the dependent variable. This consists *a* = *x* and *b* = *y*, where the sample means of *X*, *Y* are the variables *x*, *y* and the modified example standard deviations of *X* and *Y* are *sx* and *sy*, respectively.

(6) $$\begin{array}{c} r_{xy}=\frac{\sum_{i=1}^{n}\left(x_{i}-x^{`}\right)\left(y_{i}-y^{`}\right)}{\left(n-1\right)S_{x}S_{y}}=\frac{\sum_{i=1}^{n}\left(x_{i}-x^{`}\right)\left(y_{i}-y^{`}\right)}{\sqrt{\sum_{i=1}^{n}{\left(x_{i}-x`\right)}^{2}}\sum_{i=1}^{n}{\left(y_{i}-y`\right)}^{2}}. \end{array}$$

Equivalent expression *r* is calculated as follows:

(7) $$\begin{array}{c} r_{xy}=\frac{\sum x_{i}y_{i}-n\bar{x}\bar{y}}{ns_{x}^{\prime }s_{y}^{\prime }}=\frac{n\sum x_{i}y_{i}-\sum x_{i}\sum y_{i}}{\sqrt{n\sum x_{i}^{2}-{\left(\sum x_{i}\right)}^{2}}\sqrt{n\sum y_{i}^{2}-{\left(\sum y_{i}\right)}^{2}}}. \end{array}$$

The results of the measurements that contain measurement errors are *x* and *y*, and the realistic limits on the coefficient correlation are of a smaller range but not −1 to +1. The coefficient of determination was found to be *r* square which is Pearson's product-moment coefficient, for a linear model with an independent variable. An activation function “*f*” computes fresh activation at the given time *t* + 1 from *a*_*j*_(*t*), *θ*_*j*_ and the net input *p*_*j*_(*t*) giving rise to the relation.

(8) $$\begin{array}{c} a_{j}\left(t+1\right)=f\left(a_{j}\left(t\right),p_{j}\left(t\right),\theta_{j}\right), \end{array}$$

where *f*_out_ is considered as the output function.

(9) $$\begin{array}{c} o_{j}\left(t\right)=f_{\text{out}}\left(a_{j}\left(t\right)\right). \end{array}$$

The output function is simply the identity function.

(10) $$\begin{array}{c} \min_{U^{\text{T }f=\left\|U^{\text{T}}\right.}{\left.H-T\right\|}^{2}f} \end{array}$$

The original data is the input to the first block, and other blocks' downstream adds the input and the output of the preceding blocks. Knowing the weight of the upper matrix layer *U* assumed the extra masses of the systems; it is expressed as curved optimization issue and shows the closed form solution given in Equation (10). The softmax activation function is calculated as follows:

(11) $$\begin{array}{c} y_{i}=\frac{e^{x_{i}}}{\sum_{j=1}^{c}e^{x_{i}}}. \end{array}$$

The enhanced ANN is shown in Figure 3. The sparse representation fundamentally used to diminish the time complexity. In this exertion, enhanced artificial neural network result analysis has been expected to start with; at that point to surmised noisy features, a standard is set up, and finally, another enhanced artificial neural network with sparse representation classification method is anticipated. In enhanced artificial neural network, modified artificial neural network output analysis, a standard to assess the noisy features, is exhibited, which results in *m* classification for effective output

The proposed enhanced artificial neural network can be characterized in the following consequent processes:

- The realistic features are trained and forwarded by the learning stage of enhanced artificial neural network, and then, the trained enhanced artificial neural network was constant with all the factors
- By training the enhanced artificial neural network, acquire the testing feature yields
- Assess the yield by methods of the variations among the first and second biggest entries and then with the standards to compute noisy features
- By recognizable proof of enhanced artificial neural system, distinguish the effective features and support sparse representation classifier to differentiate the noisy features. From this exertion, the prediction precision has been improved. The expected enhanced algorithm is indicated

## 4. Performance Evaluation

In the entire model, TP demonstrates the true positive rate, FP demonstrates the false positive rate, TN represents the true negative rate, and FN represents the false negative rate. These measures are evaluated separately for each feature and on average for all the test features.

(12) $$\begin{array}{c} \text{Recall}=\frac{\text{True Positive}}{\text{True Positive}+\text{False Negative}}, \end{array}$$

(13) $$\begin{array}{c} \text{Specificity range}=\frac{\text{True Negative}}{\text{False Positive}+\text{True Negative }}, \end{array}$$

(14) $$\begin{array}{c} \text{Accuracy level}=\frac{\text{True Negative}+\text{True Positive}}{\text{False Negative}+\text{True Positive}+\text{False Positive}+\text{True Negative}}, \end{array}$$

(15) F‐measure=Pr·RePr+Re,

(16) $$\begin{array}{c} \text{Precision value}=\frac{\text{True Positive}}{\text{False Positive}+\text{TruePositive}}, \end{array}$$

(17) $$\begin{array}{c} \text{Sensitivity range}=\frac{\text{True Positive}}{\text{False Negative}+\text{True Positive}}. \end{array}$$

## 5. Result Analysis and Discussion

The below phase evaluated the performance of projected improved gene expression program (IGEP) with enhanced artificial neural network (EANN) process of feature selection, and the results are compared with existing algorithms like machine learning (IELM+LDA) and MRMR with support vector machine (MRMR+SVM). To estimate the survivor's time of our method, the Kaplan-Meier curve performance measure has been used. It can be measured by using the given formula.

(18) $$\begin{array}{c} \hat{N}\left(\hat{S}\left(t\right)\right)={\left(\overset{\wedge }{S}\left(t\right)\right)}^{2}\underset{i:t_{i}\leq t}{\sum }\frac{c_{i}}{n_{i}\left(n_{i}-c_{i}\right)}. \end{array}$$

The proposed schemes effectually separate the long-time survivors and short-time survivors, due to effectual optimization.  Figure 4 represents the long- and short-time survivors by class prediction using the Kaplan-Meier curve of brain cancer prognosis prediction and its comparison table in Table 3.

Figure 5 shows the ROC curve graphical representation of all methods like the proposed IGEP+EANN and existing methods like FO+GRNN, LDA+IELM, and MRMR+SVM. It illustrates the AUC of our proposed scheme that attained better value compared than other methods. These values are aligned in Table 4.

In Table 5, comparison of TP rate is mentioned and it is better than the existing scheme.

The accuracy level of proposed scheme is illustrated in Table 6.

From Figure 6, the accuracy rate of IGEP+EANN is increased better than FO+GRNN, LDA+IELM, and MRMR+SVM. Due to the effectual feature selection and retrieval, useful information by using sparse representation the TP rate has been increased, so the presented FO+GRNN attained better accuracy result. It is arranged in Tables 5 and 6. When the number of features is increased, accuracy of every scheme has been increased, due to the reduction of noisy features.

From Figure 7 and Table 7, the sensitivity rate of IGEP+EANN is decreased better than FO+GRNN, LDA+IELM, and MRMR+SVM. Due to the less error rate and true negative rate, the presented IGEP+EANN attained a better sensitivity result. The increase in the feature number increases the sensitivity, due to the high false positive rate. Compared to all algorithms, the SVM attained high sensitivity, due to the high error rate.

From Figure 8 and Table 8, the specificity rate of IGEP+EANN is 1.87% and 2.4%, which is increased better than FO+GRNN, LDA+IELM, and MRMR+SVM. The effectual feature reduction with effectual sparse representation and classification has reduced the error rate and increased the true positive rate, so the presented IGEP+EANN attained better specificity result.

From Figure 9 and Table 9, the precision rate of IGEP+EANN is increased better than FO+GRNN, LDA+IELM, and MRMR+SVM. Due to the specificity of high true positive rate, the presented LDA+IELM attained higher precision result compared than other algorithms. Less training time of IELM has increased the prediction accuracy through classifying more number of features with less error rate.

From Figure 10 and Table 10, the recall rate of IGEP+EANN is increased better than FO+GRNN, LDA+IELM, and MRMR+SVM. Due to high precision, specificity, and the recall rate of the proposed scheme is more efficient than existing algorithms. The proposed IGEP+EANN scheme's six volume metric results are evaluated for the TCGA dataset, and their mathematical evaluation is defined in Table 11. It demonstrates that the proposed IGEP+EANN results achieve higher performance when compared to the existing FO+GRNN, LDA+IELM, and MRMR+SVM.

The entire method's performance analysis is shown in Figure 11. All the 22 patients are correctly predicted. The effectual feature selection and sparse representation based on noisy feature reduction are used to improve the classification accuracy.

## 6. Conclusion

In this paper, IGEP with EANN-based new bioinformatics approach has been proposed to predict brain cancer cell prognosis. As said by our study, the EANN method has improved the accuracy of GBM prognosis when joining data from various sources compared to existing bioinformatics approaches. Future work includes further classification methods like the recognition of the sequence and the pattern, sequential decision-making, and the detection of novelty. The data processing mechanisms include clustering, filtering, compression, and blind source separation. Robotics embraces prostheses and the directing manipulator. Control specifies the computer numerical control.

## Figures and Tables

**Figure 1:** Static order dataset predicting dynamic order brain cancer cell.

**Figure 2:** Confusion matrix for artificial binomial terms.

**Figure 3:** Enhanced artificial neural network.

**Figure 4:** Long- and short-time survivors class prediction by using the Kaplan-Meier curve of brain cancer prognosis prediction.

**Figure 5:** Area under the curve performance.

**Figure 6:** Accuracy performance comparison.

**Figure 7:** Sensitivity performance comparison.

**Figure 8:** Specificity performance comparison.

**Figure 9:** Precision performance comparison.

**Figure 10:** Recall performance comparison.

**Figure 11:** Overall performance prediction.

**Algorithm 1:** 

**Table 1:** Comparison table for existing methods.

Methods	Pros	Cons
Logistic regression	Good performance for small-scale datasets and outputs produces for the interpreted probability	Assumptions about the data are required and provide the linear solutions
KNN	Intuitive methods	No. of neighbors are user-defined-based
SVMs	Provides the solutions for the nonlinear applications	Requires the knowledge using the kernel employment
Decision tree	Able to handle the categorical features and tune for the few parameters and performs well for huge number of features	Ensemble of interpretability is questioned

**Table 2:** Dataset.

Total population of primary	*N* = 276
Valid population	*N* = 211
Gender	Males 164, females 112
Long-time term survivors	171
Short-time term survivors	40
Median age at diagnosis	59
Median KPS	80
Median survival	386 days

**Table 3:** Statistical dataset properties.

Data category	Number	Feature number
Gene methylation	12440	53
Gene expression	17931	75
Copy number	16133	7
miRNA expression	534	5

**Table 4:** Evaluation of long-time survivors and short-time survivors.

Years	Long-time survivors	Short-time survivors
0	5.5	2.4
1000	4.3	2
2000	4.4	1.8
3000	4.5	1.8
4000	5	1.8

**Table 5:** Comparison between presented scheme and existing scheme.

%	IGEP+EANN	FO+GRNN	LDA+IELM	MRMR+SVM
0	3	2	1	0.4
0.2	3.5	2.5	2	1
0.4	4.5	3	2.5	1.5
0.6	5.5	3.5	2.9	1.9
0.8	7	4	3	2.2

**Table 6:** Accuracy comparison among all feature selection and classification schemes.

%	IGEP+EANN	FO+GRNN	LDA+IELM	MRMR+SVM
20	91	89	85	81
40	92	90	87	82
60	93	91	89	83
80	94	92	90	84
100	95	93	91	85
120	96.37	94.36	92.35	88.22

**Table 7:** Sensitivity comparison among all feature selection and classification schemes.

%	IGEP+EANN	FO+GRNN	LDE+IELM	MRMR+SVM
20	65	70	86	91
40	70	75	89	94
60	79	85	90	95
80	81	88	92	96
100	85	90	95	97
120	98.37	96.36	93.35	96.23

**Table 8:** Specificity comparison among all feature selection and classification schemes.

%	IGEP+EANN	FO+GRNN	LDE+IELM	MRMR+SVM
20	91.2	82	75	60
40	92.5	85	79	65
60	93.2	88	80	75
80	94.3	90	85	80
100	95.41	92	90	85
120	96.37	94.36	92.35	89.95

**Table 9:** Precision comparison among all feature selection and classification schemes.

%	IGEP+EANN	FO+GRNN	LDE+IELM	MRMR+SVM
20	73	69	30	20
40	72	70	40	35
60	74	72	50	45
80	75	74	60	55
100	77	75	74	72
120	78.78	77.78	76.77	70.85

**Table 10:** Recall comparison among all feature selection and classification schemes.

%	IGEP+EANN	FO+GRNN	LDE+IELM	MRMR+SVM
20	59	50	40	20
40	60	53	43	30
60	61	55	53	45
80	62	59	55	50
100	63.3	60	59	55
120	64.29	62.27	60.25	56.89

**Table 11:** Mathematical evaluation of overall performance for each DA detection schemes.

Performance metrics	IGEP+EANN	FO+GRNN	LDA+IELM	MRMR+SVM
Accuracy	96.37	94.36	92.35	88.22
Sensitivity	98.37	96.36	93.35	96.23
Specificity	96.37	94.36	92.35	89.95
Precision	78.78	77.78	76.77	70.85
Recall	64.29	62.27	60.25	56.89
*F*-measure	80.22	72.27	69.25	65.35

## Data Availability

The datasets used and/or analyzed during the current study are available from the corresponding authors on reasonable request.
